This article has been retracted.

# Evaluation of Achilles Tendon in Patients with Diabetic Foot Ulcer by High-Frequency Ultrasound Combined with Real-Time Shear-Wave Elastography

**DOI:** 10.1155/2022/4866240

**Published:** 2022-01-28

**Authors:** Fan Zhang, Juan Wang, Yulin Ma, Yi Wang, Wengang Wang, Yueheng Wang

**Affiliations:** The Second Hospital of Hebei Medical University, Ultrasonic Department, Shijiazhuang City, Hebei Province, China

## Abstract

To our best knowledge, no study investigated the utility of the combination of high-frequency US and real-time shear wave elastography (RTSWE) in the evaluation of Achilles tendon (AT). Our study aimed to evaluate AT in patients with diabetic foot ulcers using high-frequency US and RTSWE. We retrospectively reviewed 100 patients who visited our hospital due to diabetes. Patients were divided into the study group (those with diabetic foot ulcers) and the control group (those without diabetic foot ulcers). Patients' demographics, basic medical records, and laboratory tests were reviewed. High-frequency ultrasound and RTSWE were performed in both AT for all 100 patients. Young's modulus was measured at the upper, middle, and lower parts of each AT by RTSWE. There were 50 patients with diabetic foot ulcers. Patients in the study group had older age, a higher incidence of insulin use, and a higher level of cholesterol than those in the control group. However, thickness and Young's modulus of AT were comparable in two groups, when evaluated by the combination of high-frequency ultrasound and RTSWE. There was no significant difference in thickness and elastic modulus of AT in patients with and without diabetic foot ulcers when evaluated by the combination of high-frequency ultrasound and RTSWE.

## 1. Introduction

Diabetic foot is a terrible and serious complication of diabetes, which can lead to increased mortality and disability [1]. Many factors contribute to diabetic foot ulcers, including neuropathy, trauma, and peripheral artery disease [2–4]. Moreover, due to hyperglycemia, glycosylated end-products accumulate in the tissue and obstruct its normal metabolic function [5], which may make the condition worse. Tendon is one of the most vulnerable tissues in patients with diabetes, and the previous study has reported that the altered function of the tendon may contribute to the development of diabetic foot ulcer [6].

Achilles tendon (AT) is the largest tendon in the body and plays an important role in human movement. AT carries the body's largest load, stretching up to 10 times body weight during running, jumping, and hopping [7]. However, recent studies indicated that structural changes and altered stiffness in diabetic patients may increase the foot load and accelerate the occurrence of diabetic foot [8, 9]. In clinical practice, because the AT is thick and superficial, it is easy to examine its thickness and stiffness in patients with diabetes.

There is a lot of evidence that AT thickness increases in patients with diabetes [10, 11], but the data on stiffness is uncertain. Ultrasound (US) is useful for measuring mechanical of soft tissue, but the utility of US is limited in tendons [12]. Recently, several studies suggested that shear wave elastography (SWE) was a promising way to assess tissue stiffness [13]. In SWE, the US probe can generate a single shear wave across the tissue. Compared with quasistatic elastography, the SWE can calculate the elastic modulus by collecting information about the velocity as it passes through soft tissue [14]. In this way, we can examine the stiffness of AT by calculating the elastic modulus.

However, to the best of our knowledge, no study investigated the utility of the combination of high-frequency US and real-time (RT) SWE in the evaluation of AT. Our study aimed to evaluate the AT in patients with diabetic foot ulcers using high-frequency US and RTSWE.

## 2. Methods

After receiving the Institutional Review Board approval, we retrospectively reviewed patients who visited our hospital due to diabetes from January 2019 to January 2020. The diagnosis of diabetes was following the criteria of the American Diabetes Association [13]. The inclusion criteria were (1) fasting blood glucose ＞7.0 mmol/L; (2) without other systemic diseases.

The exclusion criteria were as follows: (1) patients with rheumatic disease or peripheral artery disease, (2) patients with Achilles tendinitis because of excessive movement, and (3) trauma or injury in the lower extremity. Based on the aforementioned criteria, 100 patients were included in our study. The diagnosis of diabetic foot ulcer referred to a previous study, which combined physical examination, neuropathy testing, and invasive evaluation of artery insufficient [15]. According to the presence or absence of diabetic foot ulcers, patients were divided into the study group (those with diabetic foot ulcers) and the control group (those without foot ulcers).

We manually reviewed the medical record in detail, which included patients' demographics (including sex, age, and body mass index (BMI)), basic medical information (including systolic and diastolic blood pressure, duration of diabetes, drug use, and neuropathy), and laboratory tests (including fasting plasma glucose (FPG), HbA1c%, cholesterol, triglycerides, and urinary albumin).

High-frequency ultrasound and RTSWE were performed in both AT for all 100 patients. Sonographic examinations were performed with Aixplorer diagnostic ultrasonographic system (Supersonic Imagine, France). A SuperLinear^TM^ SL15-4 linear probe with a frequency range of 4–15 MHz was used for both the conventional ultrasonographic and elastographic examinations. All sonographic examinations were performed by a radiologist with 5 years of experience in ultrasonography and elastography. We measured anteroposterior diameter in the middle portion of AT, about 2–6 cm above the calcaneal, which is the most vulnerable place in diabetic patients [13]. In the same place, we switched the ultrasonographic system into elastographic mode. The probe was placed vertically on the skin without additional pressure, and tendons were examined in the longitudinal plane. After the image is stabilized, the probe stays at the same location for three to five seconds. Young's modulus was measured at the upper, middle, and lower parts of each Achilles tendon by RTSWE. Three measurements were performed at each of the upper, middle, and lower parts, and the mean results were recorded.

Categorical data were presented as absolute value and percentage, and numerical data were presented as absolute value and percentage. The comparison of demographic and clinical characteristics between groups was conducted. For continuous variables, the student's *T*-test was used when they were in line with normal distribution, and Mann–Whitney test was used when they were not. The Chi-square test or Fisher's exact test was used for categorical variables. A *p* value less than 0.05 is considered significant. Statistical analysis was performed using SPSS version 20 (SPSS Inc., Chicago, Illinois).

## 3. Results

### 3.1. Patients' Demographics and Medical Characteristics

Demographics and medical characteristics of the two groups are compared in Table 1. There were 3 patients with and 11 patients without diabetic foot ulcers. The mean age was older in the study group (70.3 ± 2.1 years) than that in the control group (50.7 ± 16.8 years; *P* = 0.001). There were 23 (46.0%) men in the control group and 16 (32.0%) man in the study group (*P* = 0.151). The mean BMI was 25.4 ± 4.6 kg/m^2^ in the study group and 24.6 ± 2.6 kg/m^2^ in the control group (*P* = 0.707). There was no significant difference in systolic and diastolic blood pressure between the two groups. 40 (80.0%) patients in the study group used insulin and 38 patients (76.0%) used oral hypoglycemic drugs, while 32 (64.0%) patients used insulin and 37 (74.0%) used oral hypoglycemic drugs in the control group. Moreover, 41 (82.0%) patients in the study group had neuropathy, compared to 32 (64.0%) patients in the control group.

### 3.2. Comparison of Laboratory Tests in Two Groups

The mean FPG was 12.3 ± 1.5 mmol/L in the study group and 12.0 ± 4.8 mmol/L in the control group (*P* = 0.674). The mean HbA1c% was 8.0 ± 1.1 in the study group and 8.2 ± 2.4 in the control group (*P* = 0.593). There was significant higher cholesterol in the study group (2.2 ± 0.5 mg/dL) than that in the control group (3.6 ± 1.8 mg/dL; *P* = 0.007). However, there was no significant difference in mean triglycerides (*P* = 0.481). 17 (34.0%) patients in the study group and 14 (28.0%) patients in the control group had urinary albumin. A comparison of the laboratory is shown in Table 2.

### 3.3. Comparison of Thickness and Young's Modulus of AT in Two Groups

The thickness and Young's modulus of AT are compared in Table 3 and Figure 1. There was no significant difference in thickness and Young's modulus in any part of AT. In left AT, the mean thickness was 6.0 ± 0.5 mm in the study group and 5.9 ± 0.4 mm in the control group (*P* = 0.272). In right AT, the mean thickness was 6.0 ± 0.4 mm in the study group and 5.9 ± 0.4 mm in the control group (*P* = 0.272). About the elastic, in the upper parts of left AT, the mean Young's modulus was 392.8 ± 25.1 kPa in the study group and 383.5 ± 27.1 kPa in the control group (*P* = 0.085). In the middle parts of left AT, the mean Young's modulus was 374.3 ± 16.4 kPa in the study group and 370.3 ± 26.0 kPa in the control group (*P* = 0.360). In the lower parts of left AT, the mean Young's modulus was 344.7 ± 19.3 kPa in the study group and 344.5 ± 25.8 kPa in the control group (*P* = 0.965). In the upper parts of right AT, the mean Young's modulus was 408.5 ± 18.1 kPa in the study group and 398.5 ± 19.5 kPa in the control group (*P* = 0.090). In the middle parts of right AT, the mean Young's modulus was 380.4 ± 23.2 kPa in the study group and 377.7 ± 11.0 kPa in the control group (*P* = 0.269). In the lower parts of right AT, the mean Young's modulus was 340.6 ± 17.1 kPa in the study group and 335.0 ± 18.9 kPa in the control group (*P* = 0.123).

## 4. Discussion

Previous studies have suggested that the accumulation of nonenzymatic glycation in diabetic patients can lead to structural reorganization [16]. In animal models, hyperglycemia was found to be associated with a significant decrease in maximum load, tensile stress, stiffness, and elastic modulus of AT [17, 18].

In our study, we used a novel technique (RTSWE) to measure the elastic modulus of AT (see Figure 2). The previous study has validated the utility of SWE in measuring viscoelastic properties of tendons by comparing the wave speed of SWE with magnetic resonance imaging in agarose gels of different concentrations. This study found that SWE was a promising way to detect the change of elastic modulus in the injury and recovery period of AT [12]. Compared with other methods for the detection of AT, RTSWE has two advantages. First, the excitation frequency may be over the upper limit of commercial systems in normal AT, but RTSWE can eliminate this weakness with the use of high-frequency ultrasound. In addition, RTSWE is simple to use. Clinicians only need to adjust the machine mode without additional work. Therefore, it is feasible to evaluate AT in patients with diabetic foot ulcers as well as health AT using the combination of RTSWE and high-frequency ultrasound.

Our study found that there was no significant difference in either thickness or Young's modulus of AT between patients with and without diabetic foot ulcers. Our results were consistent with some previous literature studies [19, 20]. Giacomozzi et al. studied 61 diabetic patients with and without neuropathy and 21 healthy volunteers. They found that thickness of AT was significantly higher in diabetic patients than in healthy volunteers, but no significant difference was found in diabetic patients with and without neuropathy. In addition, they found that the flexion degree was higher in healthy volunteers, but there was still no difference in diabetic patients with and without neuropathy. This study also suggested that the duration of diabetes and comorbidities can influence the thickness of AT [19]. D'Ambrogi et al. suggested that AT was significantly thicker in patients with neuropathy, but it has begun to appear in many diabetic patients without neuropathy [20]. Moreover, previous studies also found HbA1c levels were associated with the thickness of AT [13, 17]. In our study, we divided patients into patients with and without diabetic foot ulcers, but the incidence of neuropathy and HbA1c levels were similar in the two groups. This may explain why there was no significant difference in thickness and Young's modulus between the two groups. In addition, the size of samples was relatively low in our study, which may be insufficient to make conclusions.

There were several limitations in our studies. First, this was a retrospective study, and the inherent bias cannot be avoided. Though we reviewed the medical data in detail, some mistakes may still exist. Second, the sample size of our study was quite small, which may influence the validation of our results. Further studies with a larger sample size are needed to validate the results.

## 5. Conclusion

In conclusion, there was no significant difference in thickness and elastic modulus of AT in patients with and without diabetic foot ulcers, when evaluated by the combination of high-frequency ultrasound and RTSWE.[21].

## Figures and Tables

**Figure 1:** A high-frequency ultrasound was used to detect AT. (a) Longitudinal section of normal AT. (b) Cross section of normal AT. The two-dimensional cross section of the normal AT shows oval or elliptical tendon echoes, and the boundary between the AT and the surrounding soft tissues is clear; there is no fluid accumulation in the posterior calcaneal bursa, and no calcification at the calcaneal attachment. (c) Longitudinal section of AT in diabetic patients. The tendon fibres are still running clear, and there is calcification at the calcaneal attachment. (d) Cross section of AT in diabetic patients. AT is thicker than healthier.

**Figure 2:** RTSWE was used to detect AT. (a) The elastic chart of the upper part of the normal AT is mainly yellow, with a little red. (b) The elastic chart of the middle part of the normal AT is mainly green, with a little yellow in between. (c) The elastic chart of the lower part of the normal AT is mainly blue, with a little green in between. (d) The elastic chart of the upper part of the diabetic AT is mainly red, with a little green in between. (e) The elastic chart of the middle part of the diabetic AT is mainly yellow, with a little green in between. (f) The elastic chart of the lower part of the diabetic AT is mainly yellow, with a little green in between.

**Table 1:** Demographics and medical characteristics of two groups.

	Study group (*n* = 50）	Control group（*n* = 50）	*P* value
Age (years)	70.3 ± 2.1	50.7 ± 16.8	0.001

*Sex*			0.151
Man	23 (46.0%)	16 (32.0%)	
Woman	27 (54.0%)	34 (68.0%)	

BMI (kg/m^2^)	25.4 ± 4.6	24.6 ± 2.6	0.746
Systolic blood pressure (mmHg)	122.7 ± 10.6	121.5 ± 14.4	0.636
Diastolic blood pressure (mmHg)	83.0 ± 11.9	81.3 ± 13.8	0.511
Duration of diabetes (months)	20.3 ± 12.7	5.9 ± 5.0	<0.001

*Drug use*			
Insulin	40 (80.0%)	32 (64.0%)	0.075
Oral hypoglycemic drugs	38 (76.0%)	37 (74.0%)	0.817
Neuropathy	41 (82.0%)	32 (64.0%)	0.043

**Table 2:** Comparison of laboratory tests in two groups.

	Study group （*n* = 50）	Control group （*n* = 50）	*P* value
FPG (mmol/L)	12.3 ± 1.5	12.0 ± 4.8	0.674
HbA1c (%)	8.0 ± 1.1	8.2 ± 2.4	0.593
Cholesterol (mg/dL)	2.2 ± 0.5	3.6 ± 1.8	0.007
Triglycerides (mg/dL)	1.9 ± 0.6	1.8 ± 0.8	0.481
Presence of urinary albumin	17 (34.0%)	14 (28.0%)	0.517

**Table 3:** Comparison of thickness and Young's modulus of AT in two groups.

	Study group （*n* = 50）	Control group （*n* = 50）	*P* value
*Thickness (mm)*			
Left AT	6.0 ± 0.5	5.9 ± 0.4	0.272
Right AT	6.0 ± 0.4	5.9 ± 0.4	0.214

*Young's modulus (kPa)*			
Upper parts of left AT	392.8 ± 25.1	383.5 ± 27.1	0.085
Middle parts of left AT	374.3 ± 16.4	370.3 ± 26.0	0.360
Lower parts of left AT	344.7 ± 19.3	344.5 ± 25.8	0.965
Upper parts of right AT	408.5 ± 18.1	398.5 ± 19.5	0.090
Middle parts of right AT	380.4 ± 13.2	377.7 ± 11.0	0.269
Lower parts of right AT	340.6 ± 17.1	335.0 ± 18.9	0.123

## Data Availability

The data used to support this study are available from the corresponding author upon request.
